The article "Economic Order Quantity Model with Weibull Distributed Deterioration under a Mixed Cash and Prepayment Scheme" was published in 2021. Journal: Comput Intell Neurosci.

# Economic Order Quantity Model with Weibull Distributed Deterioration under a Mixed Cash and Prepayment Scheme

**DOI:** 10.1155/2021/9588685

**Published:** 2021-09-04

**Authors:** Huda M. Alshanbari, Abd Al-Aziz H. El-Bagoury, Md. Al-Amin Khan, Soumen Mondal, Ali Akbar Shaikh, Abdur Rashid

**Affiliations:** ^1^Department of Mathematical Sciences, College of Science, Princess Nourah bint Abdulrahman University, Riyadh, Saudi Arabia; ^2^Department of Mathematics, Faculty of Science, Tanta University, Tanta, Egypt; ^3^Department of Mathematics, Jahangirnagar University, Savar, Dhaka 1342, Bangladesh; ^4^Department of Mathematics, The University of Burdwan, Burdwan 713104, India

## Abstract

Two distinct inventory models are investigated for a deteriorating item under the frequency of advertisement and market price-sensitive aggregate demand where the deterioration percentage complies with Weibull distribution. In one model, the stock-out environment is not studied, while another one handles the stock-out situation by moderately backordering based upon the waiting time duration for the products. Advance payment, another realistic feature, is implemented by paying off a fraction of the acquisition cost amid single or many equal segments from the order placing moment to receiving moment whereas the remaining fraction is accomplished at the order delivery instant by the practitioner to the supplier. The utmost aim is computing the inventory policy along with the market price and marketing strategy to reach the highest total profit for both models. The models formulated here extend several inventory studies previously developed in the literature and suggest several important outcomes. This makes two exceedingly nonlinear and mixed-integer optimization problems, which are elucidated by constructing two efficacious algorithms. Two numerical illustrations are accomplished to perceive the working competence of the algorithms and the consequences of the parameters on the practitioner's optimal policy are highlighted in a tabular form executing a sensitivity examination. Based on the performed analyses, finally, some decision-making salient findings are obtained.

## 1. Introduction

In the inventory literature, a plethora of research studies have been reported by quite a lot of researchers in the related area/field of permissible delay in payments whereas very few research works have been studied taking into consideration of advance payment scheme. Advance payment scheme ensures payment as well as delivering the goods on time. The conception of early payment was introduced in a study of Zhang [1]. In his model, he considered a fixed per-payment cost. After a long time, Maiti et al. [2] investigated an inventory system with prepayment effect. Gupta et al. [3] proposed another model taking all the parameters into interval-value under early payment scheme, solved by genetic algorithm. Thangam [4] studied an advance payment inventory model employing a discount on market price for a decay product. Taleizadeh et al. [5] investigated a model with multiple prepayments under constant demand while Zhang et al. [6] studied inventory models adopting early payment in one model and both early payment and delayed payment in another model. Taleizadeh [7] introduced a model which handles evaporating items incorporating an early payment system. Taleizadeh [8] modified Taleizadeh [7] by taking multiple prepayments with partially backlogged shortages. Afterward, Zia and Taleizadeh [9] established a model by taking both early payment and delayed payment together whereas Zhang et al. [10] suggested another model to study a supply chain environment integrating the early payment system. Li et al. [11] investigated cash flow analysis for deteriorating inventory model under advance payment scheme. Taleizadeh [12] studied the disruption effect in the inventory system with advance payment situations. Khan et al. [13] and Khan et al. [14] investigated the consequences of multiple prepayment system taking account of capacity limitation of the practitioner's warehouse. Shaikh et al. [15] presented an early payment model assuming all parameters in interval type to reflect the impreciseness. Khan et al. [16] and Rahman et al. [17] allowed a discount opportunity against prepayment scheme while Khan et al. [18] permitted a decreasing prepayment option scheme according to the purchase product amount.

The article "Economic Order Quantity Model with Weibull Distributed Deterioration under a Mixed Cash and Prepayment Scheme" was published in 2021. Journal: Comput Intell Neurosci.

Advertisement of the product is the key factor to know about the product details and hence, it has direct consequences on the market demand of that product. The practitioners/retailers have desire to broadcast the advertisements for the product to inform about the key features of the product and attract the customers in order to buy the product. Due to this circumstance, they want to use the popular electronic and print media (e.g., television, newspaper, cinema, poster, etc.). This type of concept was first introduced by Kotler [19] and he studied a model with related pricing of the product. Ladany and Sternlieb [20] proposed a selling price affected inventory model and solved it. Subramanyam and Kumaraswamy [21] studied a model integrating changeable marketing strategies while Urban [22] proposed an inventory problem with marketing decisions. Goyal and Gunasekaran [23] investigated a joined production coordination for decaying products. Shah et al. [24] formulated a model with a marketing policy for deteriorating items. Khan et al. [25] discussed the impact of marketing strategy on demand for perishable items having certain lifetime and achieved the best marketing strategy considering discrete variable. San-José et al. [26] obtained the optimal advertising policy adopting a power demand customers' demand in an inventory model.

The article "Economic Order Quantity Model with Weibull Distributed Deterioration under a Mixed Cash and Prepayment Scheme" was published in 2021. Journal: Comput Intell Neurosci.

Market price of any product is also an important issue of the market demand. When the market price of an item is high-rise, the market demand for the product is very low and vice versa. So, it has an indispensable function in inventory controlling. When a manufacturer launches a product in the market, they are acutely conscious about both the demand and market price of that product. In this connection, some extent relevant works are described. Sana [27] proposed a model for decaying items whose market demand relies upon price. Maihami and Kamalabadi [28] explored the best inventory and pricing strategies for non-instantaneous decay items under backlogging. Avinadav et al. [29] studied the deteriorating inventory model under price-sensitive demand. Ghoreishi et al. [30] described a model for the deteriorating items incorporating credit financing opportunity when market demand depends on price. Alfares and Ghaithan [31] introduced all-units reduction facility in the inventory system when market demand depends on price. Jaggi et al. [32] studied a credit supporting model assuming price-dependent market demand under two warehouse arrangements. Exploring the consequence of product lifetime on the decaying rate, Khan et al. [33] obtained the best market pricing strategy when market demand depends on price linearly. Afterward, Khan et al. [34] explored the best pricing tactic when the supplier allows a quantity based concession environment.

After certain time period every product loses its freshness and this genre of phenomenon is usually called deterioration. For the first time, Ghare and Schrader [35] proposed this genre of concept in the existing literature. Philip [36] generalized this concept and introduced Weibull distribution deterioration in the field of inventory regulation. Skouri et al. [37] inspected the consequence of ramp type market demand for a decaying item whose decay rate is characterized as a Weibull distributed function. Hung [38] modified Skouri et al. [37] model by taking partially backlogged shortages with the same type of demand. Sarkar and Sarkar [39] introduced another model where the decline rate is time-varying. Sarkar et al. [40] presented a credit financing associated model for decaying items whose rate of decay is time related. Tiwari et al. [41] studied expiration date related deteriorating inventory model under trade credit financing. Later, Shaikh et al. [42] examined the consequences of deterioration on the practitioner's purchase product amount under a quantity based concession scheme. Recently, Das et al. [43] formulated another model for decaying items allowing fractional credit financing prospect. Rana et al. [44] investigated the freshness effects on the inventory policy under limited capacity of the practitioner's storage. Duary et al. [45] investigated the consequences of both prepayment and delay payment schemes on the decision-making policy for a deteriorating item under limited storage capacity.

The article "Economic Order Quantity Model with Weibull Distributed Deterioration under a Mixed Cash and Prepayment Scheme" was published in 2021. Journal: Comput Intell Neurosci.

Taleizadeh [12], Khan et al. [14], and Rahman et al. [17] investigated the consequences of prepayment on the practitioner's best inventory strategy for decay items where the decay rate was adopted as constant. In the literature of prepayment policy in inventory management, no work has been done adopting the decay rate as two-parameter Weibull function. This work tries to cover this research gap and suggests the best management policy to the practitioner to run the business successfully under this environment.

The present work articulates two inventory problems considering the product's demand is dependent not only on price but also on number of advertisements with mixed prepayment and cash-on-delivery scheme. Moreover, the decay rate of the products obeys two-parameter Weibull function. For the first problem, no shortage is permitted while the situation with shortage is studied in the second problem where waiting time associated backlogging rate is incorporated. In addition, the supplier provides a punctual product delivery assurance against a fractional prepayment scheme where the scheme allows prepaying several equal segments instead of single installment prior to the delivery of the products. Due to discrete nature of the advertisement and Weibull distributed deterioration, both inventory problems become mined-integer nonlinear maximization problems and hence, problems are not solved analytically. To the authors' best knowledge, this work investigates the impact of mixed cash and prepayment on the optimal pricing and inventory policies for the first time when the products' deterioration follows Weibull distribution. The validity of both formulated inventory problems is examined by studying two numerical examples. As a final point, the effects of the values of the parameters are delineated after changing the values symmetrically and presenting the sensitivity analysis in a tabular form for the case with shortages, hence concluding several managerial insights for the practitioner.

The article "Economic Order Quantity Model with Weibull Distributed Deterioration under a Mixed Cash and Prepayment Scheme" was published in 2021. Journal: Comput Intell Neurosci.

## 2. Problem Explanation

This paper deliberates a three-echelon supply chain (manufacturer-retailer-customer) inventory model for a highly demandable deteriorating product (for instance, seasonal fruits, vegetables, bakeries, etc.). To retard the number of cancelling orders, manufacturer or supplier asks for a certain fraction of the purchase price prior to a fixed time interval of the received moment of the products. In return, the retailer gets an assurance for a well-timed transfer of the items whose market demand is associated with both price and the number of advertisements. Furthermore, shortages are partly backlogged depending upon the arrival time of the next delivery. This paper finds the best selling price, number of advertisements, and replenishment cycle length for maximizing the practitioner's average profit.

### 2.1. Notation

With the purpose of formulating the proposed problems, the notations given in Table 1 are utilized.

### 2.2. Assumptions

The following assumptions are taken under consideration to formulate the models:

1. Both models are fitted for a single-decay item.
2. Renewal rate is unlimited and instant.
3. A higher selling price of any product retards the customers' demand significantly whereas advertisement of any product promotes the popularity to the customers and hence proliferates the number of potential customers dramatically. Consequently, the demand pattern of the product can be considered as a linearly decreasing function of price and the exponential form of the frequency of advertisement, i.e., *D*(*A*, *p*)=*A*^*γ*^(*a* − *bp*), where *a* is the fixed demand rate, *b* is the price coefficient, *p* is the per unit selling price which is always less than (*a*/*b*), *A* is the number of advertisement, and *γ* is the advertising elasticity (0 ≤ *γ* < 1).
4. The decay rate *θ*(*t*) is increasing with respect to the elapsed time of the products in the warehouse and obeys a two-parameter Weibull distribution function of the elapsed period which can be expressed as follows: *θ*(*t*)=*αβt*^*β*−1^, where *α* ∈ (0,1) is the scale factor and *β* > 0 is the shape factor. It is noteworthy that if *β* ∈ (0,1), the deterioration rate *θ*(*t*) is suitable for the products whose deterioration rates are decreasing functions of the elapsed time whereas for *β* ∈ (1, *∞*) the deterioration rate *θ*(*t*) is suitable for the products whose deterioration rates are increasing functions of the elapsed time. Additionally, if *β*=1, then the deterioration rate becomes a constant function.
5. There is no option to return or repair a deteriorated item.
6. Shortages are fulfilled with the rate (1/1+*δu*), where *u* reveals the customers' waiting time. This takes account of the special case in which shortages are fully backlogged, which happens when *δ*=0.
7. Prepayment is accomplished by only *α*_1_ percentage of the purchase price by dint of *n* equal segments within *L* time units prior to the received moment of the products while the remaining (1 − *α*_1_) percentage is accomplished on the receiving moment of the products by the practitioner.

The article "Economic Order Quantity Model with Weibull Distributed Deterioration under a Mixed Cash and Prepayment Scheme" was published in 2021. Journal: Comput Intell Neurosci.

## 3. Model Creation

In this section, a pair of inventory problems, specifically, the inventory system where no shortage is permitted and the inventory system with shortages, are delineated mathematically by dint of the above-mentioned assumptions. Firstly the inventory system with no shortage is discussed and secondly the inventory system with shortages.

### 3.1. Inventory Procedure with No Shortage

A single-deteriorating-item inventory system is considered for a retailer where the practitioner generates an order of *Q* units by giving some portion *α*_1_ ∈ [0,1] of the purchase price *L* time units before the transfer time to his supplier. To motivate the practitioner about this prepayment, the supplier provides the opportunity to pay not at a time but by *n* identical installments at identical intervals during *L* time units. The remaining (1 − *α*_1_) percentage of the purchase price is accomplished at *t*=0. Shortly after, the products are started to be consumed to meet the demand and depleted totally at time *t*=*T* as the resulting consequences of the customers' demand and product decay. The depiction of the entire inventory procedure is provided in Figure 1.

The product level *q*(*t*) at any instant *t* during [0, *T*] obeys the following equation:

(1) $$\begin{array}{c} \frac{\text{d}q\left(t\right)}{\text{d}t}+\alpha \beta t^{\beta -1}q\left(t\right)=-D,\;0<t\leq T, \end{array}$$

with the complementary settings $q\left(t\right)=\left\{\begin{array}{cc} Q & \text{at }t=0\\ 0 & \text{at }t=T \end{array}\right.$.

The solution of equation (1), using the expansion of exponential function and *q*(*t*)=0 at *t*=*T*, is

(2) $$\begin{array}{c} q\left(t\right)\approx De^{-\alpha t^{\beta }}\left[\left(T+\frac{\alpha }{\beta +1}T^{\beta +1}+\frac{\alpha^{2}}{2\left(2\beta +1\right)}T^{2\left(2\beta +1\right)}\right)-\left(t+\frac{\alpha }{\beta +1}t^{\beta +1}+\frac{\alpha^{2}}{2\left(2\beta +1\right)}t^{2\left(2\beta +1\right)}\right)\right]. \end{array}$$

Consequently, the total number of purchase amounts *Q* for every cycle is

(3) $$\begin{array}{c} Q=q\left(0\right)\approx D\left(T+\frac{\alpha }{\beta +1}T^{\beta +1}+\frac{\alpha^{2}}{2\left(2\beta +1\right)}T^{2\left(2\beta +1\right)}\right). \end{array}$$

Then, the purchase price for every cycle is

(4) $$\begin{array}{c} PC=C_{p}Q. \end{array}$$

Since the inventory level *q*(*t*) is positive when *t* ∈ [0, *T*], consequently, the holding cost for every cycle is

(5) $$\begin{array}{c} HC=h\int_{0}^{T}q\left(t\right)\text{d}t\\ \approx h\;D\left[\frac{T^{2}}{2}+\frac{\alpha \beta T^{\beta +1}}{\left(\beta +1\right)\left(\beta +2\right)}+\frac{\alpha^{2}\left(2\beta^{2}+1\right)T^{2\beta +2}}{4{\left(\beta +1\right)}^{2}\left(2\beta +1\right)}-\frac{\alpha^{3}\beta T^{3\beta +2}}{2\left(\beta +1\right)\left(2\beta +1\right)\left(3\beta +2\right)}\right]. \end{array}$$

For each cycle, the capital cost which can be computed straightforwardly from Figure 1 is as follows:

(6) $$\begin{array}{c} CC=I_{c}\left[\frac{\alpha_{1}C_{p}Q}{n}\cdot \frac{L}{n}\left(1+2+3+\cdots +n\right)\right]=\frac{n+1}{2n}I_{c}\alpha_{1}LC_{p}Q. \end{array}$$

As the cost per advertisement to broadcast through different popular media is *G*, the advertisement cost during each cycle is

(7) $$\begin{array}{c} AC=A\cdot G. \end{array}$$

The cost to place an order is *OC*=*C*_0_.

The article "Economic Order Quantity Model with Weibull Distributed Deterioration under a Mixed Cash and Prepayment Scheme" was published in 2021. Journal: Comput Intell Neurosci.

The practitioner's total sales revenue during *t* ∈ [0, *T*] is

(8) $$\begin{array}{c} SR=p\int_{0}^{T}D\text{d}t=p\;DT\;. \end{array}$$

Hence, the profit of the practitioner in unit time is

(9) $$\begin{array}{c} Z_{1}\left(A,p,T\right)=\frac{1}{T}\left[SR-OC-AC-PC-CC-HC\right], \end{array}$$

(10) $$\begin{array}{c} =\frac{1}{T}\left[\begin{array}{c} p\;DT-C_{0}-AG-\left(1+\frac{n+1}{2n}I_{c}\alpha_{1}L\right)C_{p}D\left(T+\frac{\alpha T^{\beta +1}}{\beta +1}+\frac{\alpha^{2}T^{2\left(2\beta +1\right)}}{2\left(2\beta +1\right)}\right)\\ -h\;D\left(\frac{T^{2}}{2}+\frac{\alpha \beta T^{\beta +1}}{\left(\beta +1\right)\left(\beta +2\right)}+\frac{\alpha^{2}\left(2\beta^{2}+1\right)T^{2\beta +2}}{4{\left(\beta +1\right)}^{2}\left(2\beta +1\right)}-\frac{\alpha^{3}\beta T^{3\beta +2}}{2\left(\beta +1\right)\left(2\beta +1\right)\left(3\beta +2\right)}\right) \end{array}\right]. \end{array}$$

Now, the utmost aim is to optimize the practitioner's profit *Z*_1_(*A*, *p*, *T*) finding the best values of all decision variables, namely, number of advertisements (*A*), price (*p*), and cycle period (*T*).

The inventory system with partly backorders depending on the arrival time of the next shipment is formulated in the next section.

### 3.2. Inventory Procedure with Shortages

Here a practitioner's inventory procedure for a single-decay item, as shown in Figure 2, is considered where an order of *Q*=(*S*+*R*) units is created by paying a portion *α*_1_ ∈ [0,1] of the total purchasing price *L* time units before the transfer time to his supplier. The prepayment has to be made with *n* equal segments during *L* time units. The remaining (1 − *α*_1_) percentage of the purchase price is paid at time *t*=0, that is, order receiving moment. After receiving the products, the practitioner fulfills the amassed backorder *R* promptly and hence, the remaining stock amount in the warehouse becomes *S*. Due to the resulting consequences of the customers' demand and product decay, the number of products in the storage falls continuously and becomes empty at *t*=*t*_1_. Then, during [*t*_1_, *T*] shortages are gathered with a rate depending on the arrival time of the next shipment.

The article "Economic Order Quantity Model with Weibull Distributed Deterioration under a Mixed Cash and Prepayment Scheme" was published in 2021. Journal: Comput Intell Neurosci.

Now, the product level *q*(*t*) at any instant *t* during [0, *T*] obeys the following equations:

(11) $$\begin{array}{c} \frac{\text{d}q\left(t\right)}{\text{d}t}+\alpha \beta t^{\beta -1}q\left(t\right)=-D,\;0<t\leq t_{1}, \end{array}$$

(12) $$\begin{array}{c} \frac{\text{d}q\left(t\right)}{\text{d}t}=-\frac{D}{1+\delta \left(T-t\right)},\;t_{1}<t\leq T, \end{array}$$

with the complementary settings *q*(*t*)=*S* at *t*=0,  *q*(*t*)=0 at *t*=*t*_1_, and *q*(*t*)=−*R* at *t*=*T*.

The solutions of equations (11) and (12), using the expansion of exponential function along with *q*(*t*)=*S* at *t*=0,  *q*(*t*)=0 at *t*=*t*_1_, and *q*(*t*)=−*R* at *t*=*T*, are expressed as follows:

(13) $$\begin{array}{c} q\left(t\right)\approx De^{-\alpha t^{\beta }}\left[\left(t_{1}+\frac{\alpha t_{1}^{\beta +1}}{\beta +1}+\frac{\alpha^{2}t_{1}^{2\left(2\beta +1\right)}}{2\left(2\beta +1\right)}\right)-\left(t+\frac{\alpha t^{\beta +1}}{\beta +1}+\frac{\alpha^{2}t^{2\left(2\beta +1\right)}}{2\left(2\beta +1\right)}\right)\right],\;0<t\leq t_{1},\\ q\left(t\right)=\frac{D}{\delta }\ln\left|1+\delta \left(T-t\right)\right|-R,\;t_{1}<t\leq T. \end{array}$$

Utilizing the auxiliary condition *q*(0)=*S* at *t*=0, one has

(14) $$\begin{array}{c} S\approx D\left(t_{1}+\frac{\alpha t_{1}^{\beta +1}}{\beta +1}+\frac{\alpha^{2}t_{1}^{2\left(2\beta +1\right)}}{2\left(2\beta +1\right)}\right). \end{array}$$

The amount of total backordered quantities, adopting the continuity of *q*(*t*) at *t*=*t*_1_, is

(15) $$\begin{array}{c} R=\frac{D}{\delta }\ln\left|1+\delta \left(T-t_{1}\right)\right|. \end{array}$$

Hence, the total number of order quantities is given by

(16) $$\begin{array}{c} Q=S+R. \end{array}$$

Consequently, the purchase price during a cycle is

(17) $$\begin{array}{c} PC=C_{p}Q. \end{array}$$

As the inventory level *q*(*t*) is positive for *t* ∈ [0, *t*_1_], the cost to hold the items for a cycle is

(18) $$\begin{array}{c} HC=h\int_{0}^{t_{1}}q\left(t\right)\text{d}t\\ \approx h\;D\left[\frac{t_{1}^{2}}{2}+\frac{\alpha \beta t_{1}^{\beta +1}}{\left(\beta +1\right)\left(\beta +2\right)}+\frac{\alpha^{2}\left(2\beta^{2}+1\right)t_{1}^{2\beta +2}}{4{\left(\beta +1\right)}^{2}\left(2\beta +1\right)}-\frac{\alpha^{3}\beta t_{1}^{3\beta +2}}{2\left(\beta +1\right)\left(2\beta +1\right)\left(3\beta +2\right)}\right]. \end{array}$$

From Figure 2, the capital cost for each cycle is

(19) $$\begin{array}{c} CC=I_{c}\left[\frac{\alpha_{1}C_{p}Q}{n}\cdot \frac{L}{n}\left(1+2+3+\cdots +n\right)\right]=\frac{n+1}{2n}I_{c}\alpha_{1}LC_{p}Q. \end{array}$$

Since the cost per advertisement to broadcast through different popular media is *G*, the advertisement cost during each cycle is

(20) $$\begin{array}{c} AC=A\cdot G. \end{array}$$

As the stock becomes empty at *t*=*t*_1_, after that, shortages are performed and collected for *t* ∈ [*t*_1_, *T*] partly with a rate depending upon the arrival time of the new replenishment. Consequently, the total shortage cost for a replenishment cycle is

(21) $$\begin{array}{c} SC=C_{s}\int_{t_{1}}^{T}\left[-q\left(t\right)\right]\text{d}t\\ =\frac{C_{s}D}{\delta }\left[\left(T-t_{1}\right)-\frac{\ln\left|1+\delta \left(T-t_{1}\right)\right|}{\delta }\right]. \end{array}$$

Since the shortages are collected partly, some loses of sale occurred and the resultant cost for the lost sales is

(22) $$\begin{array}{c} \text{LSC}=c_{l}\int_{t_{1}}^{T}D\left(1-\frac{1}{1+\delta \left(T-t\right)}\right)\text{d}t\\ =C_{l}D\left[\left(T-t_{1}\right)-\frac{\ln\left|1+\delta \left(T-t_{1}\right)\right|}{\delta }\right]. \end{array}$$

The cost to generate an order is *OC*=*C*_0_. The practitioner's sales revenue during [0, *T*] is

(23) $$\begin{array}{c} SR=p\int_{0}^{t_{1}}D\text{d}t+pR=p\;DT+pR. \end{array}$$

So the profit of the practitioner in unit time is

(24) $$\begin{array}{c} Z_{2}\left(A,p,t_{1},T\right)=\frac{1}{T}\left[SR-OC-AC-PC-CC-HC-SC-LSC\right], \end{array}$$

(25) $$\begin{array}{c} =\frac{1}{T}\left[\begin{array}{c} p\;Dt_{1}+pR-C_{0}-AG-\left(1+\frac{n+1}{2n}I_{c}\alpha_{1}L\right)C_{p}Q-\left(C_{l}+\frac{C_{s}}{\delta }\right)D\left\{\left(T-t_{1}\right)-\frac{\ln\left|1+\delta \left(T-t_{1}\right)\right|}{\delta }\right\}\\ -h\;D\left\{\frac{t_{1}^{2}}{2}+\frac{\alpha \beta t_{1}^{\beta +1}}{\left(\beta +1\right)\left(\beta +2\right)}+\frac{\alpha^{2}\left(2\beta^{2}+1\right)t_{1}^{2\beta +2}}{4{\left(\beta +1\right)}^{2}\left(2\beta +1\right)}-\frac{\alpha^{3}\beta t_{1}^{3\beta +2}}{2\left(\beta +1\right)\left(2\beta +1\right)\left(3\beta +2\right)}\right\} \end{array}\right]. \end{array}$$

Now the utmost aim is to search the best number of advertisements *A*^*∗*^, price *p*^*∗*^, *t*_1_^*∗*^, and replenishment cyclic length *T*^*∗*^ for optimizing the practitioner's profit *Z*_2_(*A*, *p*, *t*_1_, *T*). In the upcoming section, the optimality along with the necessary and sufficient criterions for both inventory procedures is delineated.

The article "Economic Order Quantity Model with Weibull Distributed Deterioration under a Mixed Cash and Prepayment Scheme" was published in 2021. Journal: Comput Intell Neurosci.

## 4. Solution Method

Here, the solution process for the inventory procedure with no shortage is portrayed initially and then the same is done for the inventory procedure with shortages. There is an important note that frequency of advertisements *A* for both models is an integer type. As a result, the necessary and sufficient criterions are discussed for all other variables and the optimal number of advertisements *A*^*∗*^ is obtained by algorithmic approach for both models.

### 4.1. Inventory Procedure with No Shortage

Compute the first-order derivatives of *Z*_1_ against *p* and *T*, and then fixing the results as zero, the necessary criterions to find optimal *p*^*∗*^ and *T*^*∗*^are

(26) $$\begin{array}{c} \left(a-2bp\right)+\left(1+\frac{n+1}{2n}I_{c}\alpha_{1}L\right)C_{p}b\left(1+\frac{\alpha T^{\beta }}{\beta +1}+\frac{\alpha^{2}T^{4\beta +1}}{2\left(2\beta +1\right)}\right)\\ +hb\left(\frac{T}{2}+\frac{\alpha \beta T^{\beta }}{\left(\beta +1\right)\left(\beta +2\right)}+\frac{\alpha^{2}\left(2\beta^{2}+1\right)T^{2\beta +1}}{4{\left(\beta +1\right)}^{2}\left(2\beta +1\right)}-\frac{\alpha^{3}\beta T^{3\beta +1}}{2\left(\beta +1\right)\left(2\beta +1\right)\left(3\beta +2\right)}\right)=0, \end{array}$$

(27) $$\begin{array}{c} C_{0}+AG-\left(1+\frac{n+1}{2n}I_{c}\alpha_{1}L\right)C_{p}D\left(\frac{\alpha \beta }{\beta +1}T^{\beta +1}+\frac{\alpha^{2}\left(4\beta +1\right)}{2\left(2\beta +1\right)}T^{2\left(2\beta +1\right)}\right)\\ -h\;D\left(\frac{T^{2}}{2}+\frac{\alpha \beta^{2}T^{\beta +1}}{\left(\beta +1\right)\left(\beta +2\right)}+\frac{\alpha^{2}\left(2\beta^{2}+1\right)T^{2\beta +2}}{4{\left(\beta +1\right)}^{2}}-\frac{\alpha^{3}\beta \left(3\beta +1\right)T^{3\beta +2}}{2\left(\beta +1\right)\left(2\beta +1\right)\left(3\beta +2\right)}\right)=0. \end{array}$$

The first necessary condition, i.e., equation (26), gives

(28) $$\begin{array}{c} p=\frac{1}{2}\left[\begin{array}{c} \frac{a}{b}+\left(1+\frac{n+1}{2n}I_{c}\alpha_{1}L\right)C_{p}\left(1+\frac{\alpha T^{\beta }}{\beta +1}+\frac{\alpha^{2}T^{4\beta +1}}{2\left(2\beta +1\right)}\right)\\ +h\left(\frac{T}{2}+\frac{\alpha \beta T^{\beta }}{\left(\beta +1\right)\left(\beta +2\right)}+\frac{\alpha^{2}\left(2\beta^{2}+1\right)T^{2\beta +1}}{4{\left(\beta +1\right)}^{2}\left(2\beta +1\right)}-\frac{\alpha^{3}\beta T^{3\beta +1}}{2\left(\beta +1\right)\left(2\beta +1\right)\left(3\beta +2\right)}\right) \end{array}\right]. \end{array}$$

Using this value of *p* in equation (27) and then solving, the solution of the decision variable *T* can be found. These solutions will be optimal, if the Hessian matrix of the total profit is negative definite.

The article "Economic Order Quantity Model with Weibull Distributed Deterioration under a Mixed Cash and Prepayment Scheme" was published in 2021. Journal: Comput Intell Neurosci.

Moreover, all second derivatives against *p* and *T* are

(29) $$\begin{array}{c} \frac{\partial^{2}Z_{1}\left(.\right)}{\partial p^{2}}=-2bA^{\gamma },\\ \frac{\partial^{2}Z_{1}\left(.\right)}{\partial T\;\partial p}=A^{\gamma }\left[\begin{array}{c} \left(1+\frac{n+1}{2n}I_{c}\alpha_{1}L\right)C_{p}b\left(\frac{\alpha \beta }{\beta +1}T^{\beta -1}+\frac{\alpha^{2}\left(4\beta +1\right)}{2\left(2\beta +1\right)}T^{4\beta }\right)\\ +hb\left(\frac{1}{2}+\frac{\alpha \beta^{2}T^{\beta -1}}{\left(\beta +1\right)\left(\beta +2\right)}+\frac{\alpha^{2}\left(2\beta^{2}+1\right)T^{2\beta }}{4{\left(\beta +1\right)}^{2}}-\frac{\alpha^{3}\beta \left(3\beta +1\right)T^{3\beta }}{2\left(\beta +1\right)\left(2\beta +1\right)\left(3\beta +2\right)}\right) \end{array}\right],\\ \frac{\partial^{2}Z_{1}\left(.\right)}{\partial T^{2}}=\frac{1}{T^{2}}\left[\begin{array}{c} -\left(1+\frac{n+1}{2n}I_{c}\alpha_{1}L\right)C_{p}D\left\{\alpha \beta T^{\beta }+\alpha^{2}\left(4\beta +1\right)T^{4\beta +1}\right\}\\ -h\;D\left\{T+\frac{\alpha \beta^{2}}{\left(\beta +2\right)}T^{\beta }+\frac{\alpha^{2}\left(2\beta^{2}+1\right)}{2\left(\beta +1\right)}T^{2\beta +1}-\frac{\alpha^{3}\beta \left(3\beta +1\right)}{2\left(\beta +1\right)\left(2\beta +1\right)}T^{3\beta +1}\right\} \end{array}\right]. \end{array}$$

When eigenvalues of the corresponding Hessian matrix $\left[\begin{array}{cc} \left(\partial^{2}Z_{1}\left(.\right)/\partial p^{2}\right) & \left(\partial^{2}Z_{1}\left(.\right)/\partial p\partial T\right)\\ \left(\partial^{2}Z_{1}\left(.\right)/\partial T\partial p\right) & \left(\partial^{2}Z_{1}\left(.\right)/\partial T^{2}\right) \end{array}\right]$are negative, then the Hessian matrix of *Z*_1_ must be negative definite and hence, the solution is optimal.

Now the following set of steps is assembled to attain the best solutions of the decision variables along with the practitioner's optimal total profit.

#### 4.1.1. Algorithm to Attain the Best Solutions under the Inventory Procedure with No Shortage

 
*Step 1*. Insert the values of the parameters: *C*_0_,  *G*,  *γ*,  *C*_*p*_,  *I*_*c*_,  *h*,  *a*,  *b*,  *α*_1_,  *L*,  *n*, and initialize *Z*_1_^(max)^(*A*, *p*, *T*)=0 and *A*=1.
 
*Step 2*. Solve equation (27) for *T* adopting *p* from equation (28).
 
*Step 3.* Compute *p* from equation (28) by substituting the value of obtained *T*.
 
*Step 4*. Calculate *Z*_1_(*A*, *p*, *T*) with equation (10). If *Z*_1_(*A*, *p*, *T*) ≥ *Z*_1_^(max)^(*A*, *p*, *T*), then update the value of *Z*_1_^(max)^(*A*, *p*, *T*) by *Z*_1_(*A*, *p*, *T*) and go to Step 5. Else, toward the Step 6.
 
*Step 5.* Update *A* by *A*+1. Toward the Step 2.
 
*Step 6.* Report the best solution: *A*^*∗*^,  *p*^*∗*^,  *T*^*∗*^ and *Z*_1_^*∗*^(*A*^*∗*^,  *p*^*∗*^,  *T*^*∗*^).

The article "Economic Order Quantity Model with Weibull Distributed Deterioration under a Mixed Cash and Prepayment Scheme" was published in 2021. Journal: Comput Intell Neurosci.

### 4.2. Inventory Procedure with Shortages

Compute all the first-order derivatives of objective function *Z*_2_ against *p*,  *t*_1_, and *T*, and then fixing the results as zero, the necessary criterions to find optimal *p*^*∗*^,  *t*_1_^*∗*^, and *T*^*∗*^ are

(30) $$\begin{array}{c} \left(a-2bp\right)\left\{t_{1}+\frac{1}{\delta }\ln\left|1+\delta \left(T-t_{1}\right)\right|\right\}+b\left(C_{l}+\frac{C_{s}}{\delta }\right)\left\{\left(T-t_{1}\right)-\frac{\ln\left|1+\delta \left(T-t_{1}\right)\right|}{\delta }\right\}\\ +\left(1+\frac{n+1}{2n}I_{c}\alpha_{1}L\right)C_{p}b\left\{t_{1}+\frac{\alpha t_{1}^{\beta +1}}{\beta +1}+\frac{\alpha^{2}t_{1}^{2\left(2\beta +1\right)}}{2\left(2\beta +1\right)}+\frac{1}{\delta }\ln\left|1+\delta \left(T-t_{1}\right)\right|\right\}\\ +hb\left\{\frac{t_{1}^{2}}{2}+\frac{\alpha \beta t_{1}^{\beta +1}}{\left(\beta +1\right)\left(\beta +2\right)}+\frac{\alpha^{2}\left(2\beta^{2}+1\right)t_{1}^{2\beta +2}}{4{\left(\beta +1\right)}^{2}\left(2\beta +1\right)}-\frac{\alpha^{3}\beta t_{1}^{3\beta +2}}{2\left(\beta +1\right)\left(2\beta +1\right)\left(3\beta +2\right)}\right\}=0, \end{array}$$

(31) $$\begin{array}{c} \left(p+C_{l}+\frac{C_{s}}{\delta }\right)\left\{1-\frac{1}{1+\delta \left(T-t_{1}\right)}\right\}-\left(1+\frac{n+1}{2n}I_{c}\alpha_{1}L\right)C_{p}\left\{1+\alpha t_{1}^{\beta }+\alpha^{2}t_{1}^{4\beta +1}-\frac{1}{1+\delta \left(T-t_{1}\right)}\right\}\\ -h\left\{t_{1}+\frac{\alpha \beta t_{1}^{\beta }}{\left(\beta +2\right)}+\frac{\alpha^{2}\left(2\beta^{2}+1\right)t_{1}^{2\beta +1}}{2\left(\beta +1\right)\left(2\beta +1\right)}-\frac{\alpha^{3}\beta t_{1}^{3\beta +2}}{2\left(\beta +1\right)\left(2\beta +1\right)}\right\}=0,\\ -h\;D\left\{\frac{t_{1}^{2}}{2}+\frac{\alpha \beta t_{1}^{\beta +1}}{\left(\beta +1\right)\left(\beta +2\right)}+\frac{\alpha^{2}\left(2\beta^{2}+1\right)t_{1}^{2\beta +2}}{4{\left(\beta +1\right)}^{2}\left(2\beta +1\right)}-\frac{\alpha^{3}\beta t_{1}^{3\beta +2}}{2\left(\beta +1\right)\left(2\beta +1\right)\left(3\beta +2\right)}\right\}\\ -DT\left[\left\{p+C_{l}+\frac{C_{s}}{\delta }-\left(1+\frac{n+1}{2n}I_{c}\alpha_{1}L\right)C_{p}\right\}\frac{1}{1+\delta \left(T-t_{1}\right)}-\left(C_{l}+\frac{C_{s}}{\delta }\right)\right]=0. \end{array}$$

(32) $$\begin{array}{c} p\;Dt_{1}+pR-C_{0}-AG-\left(1+\frac{n+1}{2n}I_{c}\alpha_{1}L\right)C_{p}Q-\left(C_{l}+\frac{C_{s}}{\delta }\right)D\left\{\left(T-t_{1}\right)-\frac{\ln\left|1+\delta \left(T-t_{1}\right)\right|}{\delta }\right\}\\ -h\;D\left\{\frac{t_{1}^{2}}{2}+\frac{\alpha \beta t_{1}^{\beta +1}}{\left(\beta +1\right)\left(\beta +2\right)}+\frac{\alpha^{2}\left(2\beta^{2}+1\right)t_{1}^{2\beta +2}}{4{\left(\beta +1\right)}^{2}\left(2\beta +1\right)}-\frac{\alpha^{3}\beta t_{1}^{3\beta +2}}{2\left(\beta +1\right)\left(2\beta +1\right)\left(3\beta +2\right)}\right\}\\ -DT\left[\left\{p+C_{l}+\frac{C_{s}}{\delta }-\left(1+\frac{n+1}{2n}I_{c}\alpha_{1}L\right)C_{p}\right\}\frac{1}{1+\delta \left(T-t_{1}\right)}-\left(C_{l}+\frac{C_{s}}{\delta }\right)\right]=0. \end{array}$$

The first necessary condition, i.e., equation (30), gives the optimal selling price as

(33) $$\begin{array}{c} p=\frac{a}{2b}+\frac{\delta }{2\left\{\delta t_{1}+\ln\left|1+\delta \left(T-t_{1}\right)\right|\right\}}\left[\begin{array}{c} \left(C_{l}+\frac{C_{s}}{\delta }\right)\left\{\left(T-t_{1}\right)-\frac{\ln\left|1+\delta \left(T-t_{1}\right)\right|}{\delta }\right\}\\ +\left(1+\frac{n+1}{2n}I_{c}\alpha_{1}L\right)C_{p}\left\{t_{1}+\frac{\alpha t_{1}^{\beta +1}}{\beta +1}+\frac{\alpha^{2}t_{1}^{2\left(2\beta +1\right)}}{2\left(2\beta +1\right)}+\frac{1}{\delta }\ln\left|1+\delta \left(T-t_{1}\right)\right|\right\}\\ +h\left\{\frac{t_{1}^{2}}{2}+\frac{\alpha \beta t_{1}^{\beta +1}}{\left(\beta +1\right)\left(\beta +2\right)}+\frac{\alpha^{2}\left(2\beta^{2}+1\right)t_{1}^{2\beta +2}}{4{\left(\beta +1\right)}^{2}\left(2\beta +1\right)}-\frac{\alpha^{3}\beta t_{1}^{3\beta +2}}{2\left(\beta +1\right)\left(2\beta +1\right)\left(3\beta +2\right)}\right\} \end{array}\right]. \end{array}$$

Solving equations (31) and (32) by dint of this value of *p*, the solutions of the decision variables *t*_1_ and *T* can be obtained. These solutions will be optimal, if the Hessian matrix of the total profit is negative definite.

The article "Economic Order Quantity Model with Weibull Distributed Deterioration under a Mixed Cash and Prepayment Scheme" was published in 2021. Journal: Comput Intell Neurosci.

Now all second derivatives against *p*,  *t*_1_, and *T* are

(34) $$\begin{array}{c} \frac{\partial^{2}Z_{2}\left(.\right)}{\partial p^{2}}=-\frac{2bA^{\gamma }}{T}\left\{t_{1}+\frac{1}{\delta }\ln\left|1+\delta \left(T-t_{1}\right)\right|\right\},\\ \frac{\partial^{2}Z_{2}\left(.\right)}{\partial t_{1}\partial p}=\frac{A^{\gamma }}{T}\left[\begin{array}{c} \left\{a-2bp-b\left(C_{l}+\frac{C_{s}}{\delta }\right)\right\}\left\{1-\frac{1}{1+\delta \left(T-t_{1}\right)}\right\}\\ +\left(1+\frac{n+1}{2n}I_{c}\alpha_{1}L\right)C_{p}b\left\{1+\alpha t_{1}^{\beta }+\alpha^{2}t_{1}^{4\beta +1}-\frac{1}{1+\delta \left(T-t_{1}\right)}\right\}\\ +hb\left\{t_{1}+\frac{\alpha \beta t_{1}^{\beta }}{\left(\beta +2\right)}+\frac{\alpha^{2}\left(2\beta^{2}+1\right)t_{1}^{2\beta +1}}{2\left(\beta +1\right)\left(2\beta +1\right)}-\frac{\alpha^{3}\beta t_{1}^{3\beta +1}}{2\left(\beta +1\right)\left(2\beta +1\right)}\right\} \end{array}\right],\\ \frac{\partial^{2}Z_{2}\left(.\right)}{\partial T\;\partial p}=-\frac{A^{\gamma }}{T^{2}}\left[\begin{array}{c} \left(a-2bp\right)\left\{t_{1}+\frac{1}{\delta }\ln\left|1+\delta \left(T-t_{1}\right)\right|\right\}-b\left(C_{l}+\frac{C_{s}}{\delta }\right)\left\{t_{1}+\frac{\ln\left|1+\delta \left(T-t_{1}\right)\right|}{\delta }\right\}\\ +\left(1+\frac{n+1}{2n}I_{c}\alpha_{1}L\right)C_{p}b\left\{t_{1}+\frac{\alpha t_{1}^{\beta +1}}{\beta +1}+\frac{\alpha^{2}t_{1}^{2\left(2\beta +1\right)}}{2\left(2\beta +1\right)}+\frac{1}{\delta }\ln\left|1+\delta \left(T-t_{1}\right)\right|\right\}\\ +hb\left\{\frac{t_{1}^{2}}{2}+\frac{\alpha \beta t_{1}^{\beta +1}}{\left(\beta +1\right)\left(\beta +2\right)}+\frac{\alpha^{2}\left(2\beta^{2}+1\right)t_{1}^{2\beta +2}}{4{\left(\beta +1\right)}^{2}\left(2\beta +1\right)}-\frac{\alpha^{3}\beta t_{1}^{3\beta +2}}{2\left(\beta +1\right)\left(2\beta +1\right)\left(3\beta +2\right)}\right\}\\ -T\left\{a-2bp-b\left(C_{l}+\frac{C_{s}}{\delta }\right)+\left(1+\frac{n+1}{2n}I_{c}\alpha_{1}L\right)C_{p}b\right\}\frac{1}{1+\delta \left(T-t_{1}\right)} \end{array}\right],\\ \frac{\partial^{2}Z_{2}\left(.\right)}{\partial t_{1}^{2}}=-\frac{D}{T}\left[\begin{array}{c} \left(p+C_{l}+\frac{C_{s}}{\delta }\right)\frac{\delta }{{\left\{1+\delta \left(T-t_{1}\right)\right\}}^{2}}\\ +\left(1+\frac{n+1}{2n}I_{c}\alpha_{1}L\right)C_{p}\left\{\alpha \beta t_{1}^{\beta -1}+\alpha^{2}\left(4\beta +1\right)t_{1}^{4\beta }-\frac{\delta }{{\left\{1+\delta \left(T-t_{1}\right)\right\}}^{2}}\right\}\\ +h\left\{1+\frac{\alpha \beta^{2}t_{1}^{\beta -1}}{\left(\beta +2\right)}+\frac{\alpha^{2}\left(2\beta^{2}+1\right)t_{1}^{2\beta }}{2\left(\beta +1\right)}-\frac{\alpha^{3}\left(3\beta +1\right)\beta t_{1}^{3\beta }}{2\left(\beta +1\right)\left(2\beta +1\right)}\right\} \end{array}\right],\\ \frac{\partial^{2}Z_{2}\left(.\right)}{\partial T\;\partial t_{1}}=-\frac{D}{T^{2}}\left[\begin{array}{c} \left(p+C_{l}+\frac{C_{s}}{\delta }\right)\left\{1-\frac{1}{1+\delta \left(T-t_{1}\right)}\right\}\\ -\left(1+\frac{n+1}{2n}I_{c}\alpha_{1}L\right)C_{p}\left\{1+\alpha t_{1}^{\beta }+\alpha^{2}t_{1}^{4\beta +1}-\frac{1}{1+\delta \left(T-t_{1}\right)}\right\}\\ -h\left\{t_{1}+\frac{\alpha \beta t_{1}^{\beta }}{\left(\beta +2\right)}+\frac{\alpha^{2}\left(2\beta^{2}+1\right)t_{1}^{2\beta +1}}{2\left(\beta +1\right)\left(2\beta +1\right)}-\frac{\alpha^{3}\beta t_{1}^{3\beta +1}}{2\left(\beta +1\right)\left(2\beta +1\right)}\right\}\\ -\left\{p+C_{l}+\frac{C_{s}}{\delta }-C_{p}\left(1+\frac{n+1}{2n}I_{c}\alpha_{1}L\right)\right\}\frac{\delta T}{{\left\{1+\delta \left(T-t_{1}\right)\right\}}^{2}} \end{array}\right],\\ \frac{\partial^{2}Z_{2}\left(.\right)}{\partial T^{2}}=\frac{2}{T^{3}}\left[\begin{array}{c} p\;Dt_{1}+pR-C_{0}-AG-\left(1+\frac{n+1}{2n}I_{c}\alpha_{1}L\right)C_{p}Q-\left(C_{l}+\frac{C_{s}}{\delta }\right)D\left\{\left(T-t_{1}\right)-\frac{\ln\left|1+\delta \left(T-t_{1}\right)\right|}{\delta }\right\}\\ -h\;D\left\{\frac{t_{1}^{2}}{2}+\frac{\alpha \beta t_{1}^{\beta +1}}{\left(\beta +1\right)\left(\beta +2\right)}+\frac{\alpha^{2}\left(2\beta^{2}+1\right)t_{1}^{2\beta +2}}{4{\left(\beta +1\right)}^{2}\left(2\beta +1\right)}-\frac{\alpha^{3}\beta t_{1}^{3\beta +2}}{2\left(\beta +1\right)\left(2\beta +1\right)\left(3\beta +2\right)}\right\}\\ -DT\left[\left\{p+C_{l}+\frac{C_{s}}{\delta }-\left(1+\frac{n+1}{2n}I_{c}\alpha_{1}L\right)C_{p}\right\}\frac{1}{1+\delta \left(T-t_{1}\right)}-\left(C_{l}+\frac{C_{s}}{\delta }\right)\right]\\ -\frac{DT^{2}}{2}\left[\left\{p+C_{l}+\frac{C_{s}}{\delta }-\left(1+\frac{n+1}{2n}I_{c}\alpha_{1}L\right)C_{p}\right\}\frac{\delta }{{\left\{1+\delta \left(T-t_{1}\right)\right\}}^{2}}\right] \end{array}\right]. \end{array}$$

When eigenvalues of the corresponding Hessian matrix $\left[\begin{array}{ccc} \left(\partial^{2}Z_{2}\left(.\right)/\partial p^{2}\right) & \left(\partial^{2}Z_{2}\left(.\right)/\partial p\partial t_{1}\right) & \left(\partial^{2}Z_{2}\left(.\right)/\partial p\partial T\right)\\ \left(\partial^{2}Z_{2}\left(.\right)/\partial p\partial t_{1}\right) & \left(\partial^{2}Z_{2}\left(.\right)/\partial t_{1}^{2}\right) & \left(\partial^{2}Z_{2}\left(.\right)/\partial T\partial t_{1}\right)\\ \left(\partial^{2}Z_{2}\left(.\right)/\partial T\partial p\right) & \left(\partial^{2}Z_{2}\left(.\right)/\partial t_{1}\partial T\right) & \left(\partial^{2}Z_{2}\left(.\right)/\partial T^{2}\right) \end{array}\right]$are negative, then the Hessian matrix of *Z*_2_ must be negative definite and hence, the solution is optimal.

The article "Economic Order Quantity Model with Weibull Distributed Deterioration under a Mixed Cash and Prepayment Scheme" was published in 2021. Journal: Comput Intell Neurosci.

To attain the best solutions of the decision variables along with the practitioner's optimal profit, the following computational set of steps is proposed.

#### 4.2.1. Algorithm to Attain the Best Solutions under the Inventory Procedure with Shortages

 
*Step 1.* Insert the values of the parameters: *C*_0_,  *G*,  *γ*,  *C*_*p*_,  *I*_*c*_,  *h*,  *a*,  *b*,  *α*_1_,  *L*,  *n*,  *δ*,  *C*_*l*_,  *C*_*s*_ and initialize *Z*_2_^(max)^(*A*, *p*, *t*_1_, *T*)=0 and *A*=1.
 
*Step 2*. Solve equations (31) and (32) for *t*_1_ and *T* exploiting *p* from equation (33).
 
*Step 3.* Compute *p* from equation (33) by substituting the value of obtained *t*_1_ and *T*.
 
*Step 4*. Calculate *Z*_2_(*A*, *p*, *t*_1_, *T*) with equation (25). If *Z*_2_(*A*, *p*, *t*_1_, *T*) ≥ *Z*_2_^(max)^(*A*, *p*, *t*_1_, *T*), then update the value of *Z*_2_^(max)^(*A*, *p*, *t*_1_, *T*) by *Z*_2_(*A*, *p*, *t*_1_, *T*) and toward the Step 5. Else, toward the Step 6.
 
*Step 5*. Update*A* by *A*+1, and toward the Step 2.
 
*Step 6*. Report the best solution: *A*^*∗*^, *p*^*∗*^, *t*_1_^*∗*^, *T*^*∗*^ and *Z*_2_^*∗*^(*A*^*∗*^, *p*^*∗*^, *t*_1_^*∗*^, *T*^*∗*^).

## 5. Numerical Study

Now the applicability of the delineated inventory procedures and also several decision-making perceptions are highlighted by exploiting two numerical studies adopting the proposed computational set of steps.

**Example 1 .**

Inventory procedure with no shortage.

Consider the following data from Khan et al. [25]: *C*_0_=$500/order, *a*=250, *b*=1.9, *C*_*p*_=$50/unit, *h*=$2/unit, *α*=0.1, *β*=2, *L*=10 weeks, *n*=20, *I*_*c*_=0.05/dollar/week, *α*_1_=0.4, *γ*=0.1, *G*=$50/advertisement. With the help of the proposed computational set of steps to attain the best solutions for the inventory procedure with no shortage, the best solution is displayed in the following tabular forms.

From Table 2, the best solution is *A*^*∗*^=7, *p*^*∗*^=$95.43526, *T*^*∗*^=1.80484 weeks, *Q*^*∗*^=103.4948 units with *Z*_1_^(max)^(*A*, *p*, *T*)=$2295.240. As the eigenvalues of the Hessian matrix $\left[\begin{array}{cc} \left(\partial^{2}Z_{1}\left(.\right)/\partial p^{2}\right) & \left(\partial^{2}Z_{1}\left(.\right)/\partial p\partial T\right)\\ \left(\partial^{2}Z_{1}\left(.\right)/\partial T\partial p\right) & \left(\partial^{2}Z_{1}\left(.\right)/\partial T^{2}\right) \end{array}\right]$ are −21883.741417 and −3.691409, the obtained results are optimal. Moreover, the concavity of *Z*_1_ can be detected from Figure 3 for a fixed number of advertisements.

**Example 2 .**

Inventory procedure with shortages.

For this example, we have considered the same data that are used in Example 1 along with *δ*=1.5, *c*_*s*_=12, and *c*_*l*_=14 for the backlogged shortages. For different values of *A*, the solutions of Example 2 by dint of the proposed computational set of steps to attain the best solutions for the inventory procedure with shortages are revealed in Table 3.

Hence, the optimal solutions, from the above table, are *A*^*∗*^=8, *p*^*∗*^=$95.31335, *t*_1_^*∗*^=1.16744 weeks, *T*^*∗*^=1.33121 weeks, *S*^*∗*^=103.9339 units, *R*^*∗*^=12.42282 units, *Q*^*∗*^=116.3568 units, *Z*_2_^(max)^(*A*, *p*, *t*_1_, *T*)=$2360.342. Since the eigenvalues of the Hessian matrix $\left[\begin{array}{ccc} \left(\partial^{2}Z_{2}\left(.\right)/\partial p^{2}\right) & \left(\partial^{2}Z_{2}\left(.\right)/\partial p\partial t_{1}\right) & \left(\partial^{2}Z_{2}\left(.\right)/\partial p\partial T\right)\\ \left(\partial^{2}Z_{2}\left(.\right)/\partial p\partial t_{1}\right) & \left(\partial^{2}Z_{2}\left(.\right)/\partial t_{1}^{2}\right) & \left(\partial^{2}Z_{2}\left(.\right)/\partial T\partial t_{1}\right)\\ \left(\partial^{2}Z_{2}\left(.\right)/\partial T\partial p\right) & \left(\partial^{2}Z_{2}\left(.\right)/\partial t_{1}\partial T\right) & \left(\partial^{2}Z_{2}\left(.\right)/\partial T^{2}\right) \end{array}\right]$ are −8813.706933, −894.217364, and −4.508842, the obtained results are optimal. Moreover, the concavity of *Z*_2_ can be detected from Figures 4–6 for a fixed frequency of advertisement.

The article "Economic Order Quantity Model with Weibull Distributed Deterioration under a Mixed Cash and Prepayment Scheme" was published in 2021. Journal: Comput Intell Neurosci.

## 6. Sensitivity Analysis

To investigate the influence on *A*, *p*, *t*_1_, *T*, *S*, *R* along with the profit, a sensitivity analysis is accomplished against all the system parameters of Example 2 (shortages case) by presenting how much deviation on best values could be if each factor is innovated symmetrically in a tabular form. For this purpose, the value of each factor is changed from −20% to +20%, while the remaining factors are kept stable and the corresponding outcomes are displayed in Table 4.

Table 4 exposes that purchase quantity (*Q*^*∗*^), inventory cycle (*T*^*∗*^), and price (*p*^*∗*^) increase when the cost for placing the order increases. However, the salient thinks that the practitioner's profit decreases in this situation. Thus, a greater price does not always provide a greater profit for the decision-maker.

Both demand factors *a* and *b* have the largest consequences on the practitioner's best inventory policy and profit as well but in an opposite manner. Initial stock (*S*^*∗*^), shortages (*R*^*∗*^), price (*p*^*∗*^), and profit increase considerably when the demand factor *a* increases, while inventory cycle (*T*^*∗*^) falls because of a higher demand. On the contrary, the price coefficient *b* shows exactly opposite consequences on initial stock (*S*^*∗*^), shortages (*R*^*∗*^), price (*p*^*∗*^), inventory cycle (*T*^*∗*^), and profit as well when *b* increases.

As Table 4 shows, price (*p*^*∗*^) and inventory cycle (*T*^*∗*^) increase while purchase quantity (*Q*^*∗*^) and profit decrease when purchase price for a unit (*C*_*p*_) increases. The reason behind that is the fact that if *C*_*p*_ rises, the practitioner purchases a lower number of products and increases the market price and hence, market demand falls significantly and hence *T*^*∗*^ grows but profit shrinks.

When carrying cost for each item increases, then shortages (*R*^*∗*^) and price (*p*^*∗*^) increase but inventory cycle (*T*^*∗*^), *t*_1_^*∗*^, and profit shrink. Since the practitioner has to bear a greater carrying cost for a greater purchase amount, the practitioner makes a small order and consequently, shortages appear much more faster. Therefore, *R*^*∗*^ increases and *p*^*∗*^ increases also to cover the higher cost to hold the products.

The article "Economic Order Quantity Model with Weibull Distributed Deterioration under a Mixed Cash and Prepayment Scheme" was published in 2021. Journal: Comput Intell Neurosci.

If the advertisement elasticity (*γ*) increases, both the initial stock (*S*^*∗*^) and shortages (*R*^*∗*^) reveal an upward trend sharply. As the increment of *γ* means the positive impact of the advertisement on the market demand, practitioner enriches the initial stock amount and shortages are accumulated for a longer period with a higher demand, that is; shortages amount also enlarges significantly.

Initial stock (*S*^*∗*^), inventory cycle (*T*^*∗*^), *t*_1_^*∗*^, and profit shrink when both deterioration factors *α* and *β* grow, while shortages (*R*^*∗*^) and price (*p*^*∗*^) increase and decrease for a higher value of *α* and *β*, respectively. If *α* grows, the number of decay items also grows and hence, initial stocks decline comparatively soon and the practitioner increases *p*^*∗*^ to mitigate the loss from the deteriorated items. On the other hand, as *β* is greater than one, the number of deteriorated items is lower for a larger *β* and therefore, both shortages (*R*^*∗*^) and price (*p*^*∗*^) decrease.

The prepayment factor *n* (number of installment) has positive consequence on the practitioner's profit, while the other factors *α*_1_ (percentage to prepay) and *L* (duration to accomplish prepay) have negative consequences on the profit. When the percentage of purchase price and duration for accomplishing prepayment rise, the practitioner bears a higher cost against the capital and therefore, the profit decreases. However, for a higher *n* the practitioner creates a smaller loan and hence, he bears a higher cost against the loan for the capital.

## 7. Decision-Making Insights

Analyzing the results from the accomplished sensitivity examination, the subsequent discoveries can be exhorted to the practitioner to proliferate the profit:

- The analysis discloses that the practitioner's profit is significantly affected by the fixed demand rate parameter “*a*” and the price coefficient “*b*.” Therefore, the decision-maker is instructed to execute the appropriate marketing policies for the augmentation of the market demand.
- The demand of the product can be increased considerably by promoting products' information to the potential customers by dint of an effective advertisement telecasting through different popular media. The manager ought to create an efficacious advertisement and attempt to broadcast through different genres of media with a reasonable cost for each advertisement.
- When the number of identical segments for accomplishing prepayment at identical time intervals during the lead period rises, the practitioner's profit also rises. Hence, the decision-maker should pick the supplier offering the opportunity to prepay by a large number of identical multiple segments at identical time intervals.
- If time interval for the prepayment dwindles, then the capital cost deescalates and hence the profit also escalates. So the manager is recommended to select the supplier allowing a short lead period for accomplishing the prepayment.
- Total profit declines when the percentage of the purchase price for the prepayment increases. Therefore, it is exhorted to select the manufacturer who allows a small percentage of the purchase price for completing the prepayment.
- The purchase price for a unit item has the utmost negative influence on the practitioner's profit among all inventory related cost factors; that is, when unit purchase cost increases, the total profit decreases. Thus, decreasing purchase price for a unit item is an additional proposal for accruing the profit to the manager by discussing with the manufacturer or increasing the order size.
- When the ordering cost per order declines, the total profit escalates. So the manager is suggested to diminish the cost for creating order by increasing the purchase amount suitably.

The article "Economic Order Quantity Model with Weibull Distributed Deterioration under a Mixed Cash and Prepayment Scheme" was published in 2021. Journal: Comput Intell Neurosci.

## 8. Conclusion

This work formulates two profit optimizing inventory models (with no shortage and shortages) under a mixed cash-on and prepayment strategy for a decay product whereas the market demand of the product is associated with not only the price but also the number of advertisements through genres of media. In both cases, the optimization problems are formulated as mixed-integer optimization problems and then two algorithms are established to solve the problems. Two numerical studies are executed to examine the applicability of the proposed algorithms and also to validate the proposed models. Comparing the corresponding results it is observed that the inventory model with shortages is more economical from the profit maximizing aspect. From the analyses it is found that the decision-maker can increase profit significantly by executing the appropriate marketing policies for the augmentation of the market demand. Furthermore, the decision-maker should pick the supplier who allows the opportunity to prepay by a large number of identical multiple segments at identical time intervals during the lead time.

In future, anyone can further investigate the models by incorporating several realistic features such as nonlinear price-dependent demand pattern, stock-dependent demand, displayed stock-dependent demand, power demand pattern in time, nonlinear carrying cost, or trade credit policy. Also, relaxing the zero-ending case by nonending inventory model would be another interesting extension of the model without shortages. Moreover, considering discounts in the unit purchase price would be another interesting extension of the current models.

The article "Economic Order Quantity Model with Weibull Distributed Deterioration under a Mixed Cash and Prepayment Scheme" was published in 2021. Journal: Comput Intell Neurosci.

## Figures and Tables

**Figure 1:** Pictorial demonstration of the inventory procedure with no shortage.

**Figure 2:** Pictorial demonstration of the inventory procedure with shortages.

**Figure 3:** The concavity of *Z*_1_(*A*, *p*, *T*) for *A*=7.

**Figure 4:** The concavity of *Z*_2_ against *p* and *T* for *A*=7.

**Figure 5:** The concavity of *Z*_2_ against *T* and *t*_1_ for *A*=7.

**Figure 6:** The concavity of *Z*_2_ against *p* and *t*_1_ for *A*=7.

**Table 1:** Notation.

Symbolizations	Explanation
*C*_0_	Replenishment cost per order in dollars
*a*	Fixed demand rate (*a* > 0)
*b*	Price scale in the demand (*b* > 0)
*C*_*p*_	Purchase price ($/unit)
*p*	Price of the item ($/unit)
*θ*(*t*)	Weibull distributed decay rate (0 < *θ*(*t*) ≪ 1)
*A*	The number of advertisement
*γ*	Advertising elasticity
*G*	Cost per advertisement ($)
*h*	Holding cost ($/unit time/unit)
*C*_*s*_	Shortage cost ($/unit)
*δ*	Backlogging parameter (*δ* > 0)
*S*	Initial stock
*R*	Highest number of backorders
*Q*	Order amount (unit/order)
*C*_*l*_	Opportunity cost ($/unit)
*t*_1_	Time period of physical stock in the warehouse (time unit)
*T*	Cycle length (time unit)
*Z*_1_(*A*, *p*, *T*)	The practitioner's profit under the first inventory procedure ($/time unit)
*Z*_2_(*A*, *p*, *t*_1_, *T*)	The practitioner's profit of the inventory procedure with backorders ($/time unit)
	Decision variable
*A*	Number of advertisements
*p*	Price of the item ($/unit)
*t*_1_	Time period of physical stock in the warehouse (time unit)
*T*	Cycle length (time unit)

**Table 2:** Solution of Example 1.

*A*	*p*	*T*	*Q*	*Z*_1_(*A*, *p*, *T*)
1	95.21548	1.11614	80.52227	2019.592
2	95.23107	1.12097	86.67879	2155.136
3	95.26616	1.13174	91.13679	2221.967
4	95.30700	1.14398	94.30700	2259.549
5	95.34967	1.15644	98.01896	2280.800
6	95.39265	1.16867	100.8850	2291.628
7	**95.43526**	**1.80484**	**103.4948**	**2295.240**
8	95.47720	1.19181	105.8996	2293.576
9	95.51830	1.20263	108.1347	2287.894

Bold values indicate the optimal solutions.

**Table 3:** Solution of Example 2.

*A*	*p*	*t*_1_	*T*	*S*	*R*	*Q*	*Z*_2_(*A*, *t*_1_, *p*, *T*)
1	95.07720	1.092880	1.223702	78.98420	8.284743	87.26894	2058.742
2	95.08986	1.097667	1.230280	85.02687	8.986973	94.01385	2197.927
3	95.12171	1.108284	1.245003	89.40845	9.614820	99.02327	2268.539
4	95.15876	1.120350	1.261983	93.02806	10.20851	103.2366	2309.995
5	95.19749	1.132635	1.279563	96.17932	10.78118	106.9605	2335.205
6	95.23652	1.144682	1.297112	98.99997	11.33900	110.3390	2350.074
7	95.27523	1.156306	1.314366	101.5682	11.88546	113.4537	2357.807
8	**95.31335**	**1.167440**	**1.331210**	**103.9339**	**12.42282**	**116.3568**	**2360.342**
9	95.35075	1.178068	1.347604	106.1318	12.95262	119.0844	2358.939
10	95.38739	1.188198	1.363542	108.1870	13.47601	121.6630	2354.463

Bold values indicate the optimal solutions.

The article "Economic Order Quantity Model with Weibull Distributed Deterioration under a Mixed Cash and Prepayment Scheme" was published in 2021. Journal: Comput Intell Neurosci.

**Table 4:** Sensitivity examination of several factors on the best solution.

Parameter	Original value	% of change in the original values	% of change in					
			*t*_1_^*∗*^	*T* ^*∗*^	*S* ^*∗*^	*R* ^*∗*^	*p* ^*∗*^	Total profit
*C*_0_	500	−20	−2.59	−3.38	−2.61	−7.92	−0.11	3.24
		−10	−1.25	−1.65	−1.26	−3.94	−0.05	1.6
		10	1.16	1.58	1.17	3.91	0.05	−1.58
		20	2.25	3.09	2.27	7.79	0.1	−3.13

*a*	250	−20	4.17	11.27	−40.14	−12.9	−13.55	−72.95
		−10	1.14	3.52	−21.06	−8.04	−6.84	−41.56
		10	0.06	−1.35	23.13	10.25	6.9	52.01
		20	0.13	−2.41	46.3	18.63	13.8	114.87

*b*	1.9	−20	2.88	0.52	27.61	5.18	17.37	91.92
		−10	1.17	−0.07	13.01	2.55	7.71	39.18
		10	−0.32	1.23	−11.06	−1.06	−6.28	−29.55
		20	0.46	4.16	−19.87	0.9	−11.45	−52.06

*C*_*p*_	50	−20	3.93	1.56	24.63	2.62	−5.93	45.16
		−10	2.29	1.20	13.02	3.62	−2.95	21.52
		10	−1.18	0.35	−10.27	−0.02	2.99	−19.47
		20	−2.11	1.18	−20.04	−0.45	5.98	−36.95

*h*	2	−20	0.69	0.34	1.01	−1.75	−0.09	0.77
		−10	0.35	0.17	0.51	−0.87	−0.04	0.38
		10	−0.35	−0.17	−0.51	0.87	0.04	−0.38
		20	−0.7	−0.35	−1.01	1.73	0.09	−0.76

*α*	0.1	−20	6.56	5.46	7.62	−0.89	−0.06	2.05
		−10	2.64	1.97	2.54	−2.38	−0.05	0.98
		10	−2.36	−1.75	−2.28	2.23	0.04	−0.92
		20	−4.5	−3.31	−4.34	4.34	0.08	−1.78

*β*	2	−20	4.07	3.77	4.22	0.81	0.24	−0.54
		−10	1.81	1.68	1.88	0.4	0.11	−0.26
		10	−1.47	−1.38	−1.54	−0.39	−0.09	0.24
		20	−2.69	−2.53	−2.81	−0.77	−0.18	0.46

*α*_1_	0.4	−20	0.07	−0.25	1.59	−0.85	−0.57	3.92
		−10	0.04	−0.13	0.80	−0.43	−0.29	1.95
		10	−0.03	0.13	−0.79	0.43	0.29	−1.94
		20	−0.06	0.27	−1.58	0.85	0.57	−3.86

*δ*	1.5	−20	−0.39	1.93	−0.38	19.18	−0.02	0.5
		−10	−0.18	0.88	−0.17	8.74	−0.01	0.23
		10	0.15	−0.76	0.15	−7.44	0.01	−0.2
		20	0.28	−1.41	0.27	−13.84	0.02	−0.37

*C*_*s*_	12	−20	−0.06	0.32	−0.04	2.79	−0.01	0.08
		−10	−0.03	0.16	−0.02	1.38	−0.01	0.04
		10	0.03	−0.15	0.02	−1.34	0.01	−0.04
		20	0.06	−0.31	0.04	−2.65	0.01	−0.07

*C*_*l*_	14	−20	−0.11	0.58	−0.07	5	−0.02	0.14
		−10	−0.06	0.28	−0.04	2.44	−0.01	0.07
		10	0.05	−0.27	0.03	−2.32	0.01	−0.06
		20	0.1	−0.52	0.07	−4.54	0.02	−0.13

*L*	10	−20	0.07	−0.25	1.59	−0.85	−0.57	3.92
		−10	0.04	−0.13	0.8	−0.43	−0.29	1.95
		10	−0.03	0.13	−0.79	0.43	0.29	−1.94
		20	−0.06	0.27	−1.58	0.85	0.57	−3.86

*I*_*c*_	0.05	−20	0.07	−0.25	1.59	−0.85	−0.57	3.92
		−10	0.04	−0.13	0.80	−0.43	−0.29	1.95
		10	−0.03	0.13	−0.79	0.43	0.29	−1.94
		20	−0.06	0.27	−1.58	0.85	0.57	−3.86

*n*	20	−20	0.00	0.02	−0.09	0.05	0.03	−0.23
		−10	0.00	0.01	−0.04	0.02	0.02	−0.10
		10	0.00	−0.01	0.03	−0.02	−0.01	0.08
		20	0.00	−0.01	0.06	−0.03	−0.02	0.15

*γ*	0.1	−20	−1.16	−1.53	−7.35	−9.70	−0.05	−4.85
		−10	−0.53	−0.70	−3.74	−4.88	−0.02	−2.56
		10	0.44	0.59	3.89	4.93	0.02	2.83
		20	1.59	2.17	10.05	14.18	0.07	5.94

*G*	50	−20	−0.48	−0.65	1.76	0.66	−0.02	2.9
		−10	−0.14	−0.18	1.05	0.74	−0.01	1.37
		10	−0.07	−0.1	−1.4	−1.57	−0.003	−1.23
		20	0.76	1.03	−0.57	1.18	0.03	−2.34

The article "Economic Order Quantity Model with Weibull Distributed Deterioration under a Mixed Cash and Prepayment Scheme" was published in 2021. Journal: Comput Intell Neurosci.

## Data Availability

No data were used to support this study.
